RETRACTED

# Angiogenesis Impairment in Diabetes: Role of Methylglyoxal-Induced Receptor for Advanced Glycation Endproducts, Autophagy and Vascular Endothelial Growth Factor Receptor 2

**DOI:** 10.1371/journal.pone.0046720

**Published:** 2012-10-03

**Authors:** Hongtao Liu, Shujie Yu, Hua Zhang, Jian Xu

**Affiliations:** Section of Endocrinology, Department of Medicine, Harold Hamm Diabetes Center, University of Oklahoma Health Sciences Center, Oklahoma City, Oklahoma, United States of America; University of Illinois at Chicago, United States of America

## Abstract

Diabetes impairs physiological angiogenesis by molecular mechanisms that are not fully understood. Methylglyoxal (MGO), a metabolite of glycolysis, is increased in patients with diabetes. This study defined the role of MGO in angiogenesis impairment and tested the mechanism in diabetic animals. Endothelial cells and mouse aortas were subjected to Western blot analysis of vascular endothelial growth factor receptor 2 (VEGFR2) protein levels and angiogenesis evaluation by endothelial cell tube formation/migration and aortic ring assays. Incubation with MGO reduced VEGFR2 protein, but not mRNA, levels in a time and dose dependent manner. Genetic knockdown of the receptor for advanced glycation endproducts (RAGE) attenuated the reduction of VEGFR2. Overexpression of Glyoxalase 1, the enzyme that detoxifies MGO, reduced the MGO-protein adducts and prevented VEGFR2 reduction. The VEGFR2 reduction was associated with impaired angiogenesis. Suppression of autophagy either by inhibitors or siRNA, but not of the proteasome and caspase, normalized both the VEGFR2 protein levels and angiogenesis. Conversely, induction of autophagy either by rapamycin or overexpression of LC3 and Beclin-1 reduced VEGFR2 and angiogenesis. MGO increased endothelial LC3B and Beclin-1, markers of autophagy, which were accompanied by an increase of both autophagic flux (LC3 punctae) and co-immunoprecipitation of VEGFR2 with LC3. Pharmacological or genetic suppression of peroxynitrite (ONOO^−^) generation not only blocked the autophagy but also reversed the reduction of VEGFR2 and angiogenesis. Like MGO-treated aortas from normglycemic C57BL/6J mice, aortas from diabetic db/db and Akita mice presented reductions of angiogenesis or VEGFR2. Administration of either autophagy inhibitor *ex vivo* or superoxide scavenger *in vivo* abolished the reductions. Taken together, MGO reduces endothelial angiogenesis through RAGE-mediated, ONOO^–^dependent and autophagy-induced VEGFR2 degradation, which may represent a new mechanism for diabetic angiogenesis impairment.

## Introduction

Angiogenesis, defined as the formation of new blood vessels out of preexisting capillaries, plays a crucial role in maintaining vascular health [1]. Angiogenesis impairment operates in the peripheral vasculature contributing to delayed wound healing, exacerbated peripheral limb ischemia, and even cardiac mortality via reduction of collateral vessel development [2]. Mechanisms underlying diabetic angiogenesis impairment are complex. Multiple molecular mechanisms have been proposed, including oxidative stress/reactive oxygen species, endothelial derangements, loss of endothelium-derived nitric oxide (NO) bioactivity, and micro RNA alterations [3]. However, it has not been completely elucidated how diabetes impairs physiological angiogenesis.

RETRACTED

VEGF receptor 2 (VEGFR2, or kinase-insert domain receptor, KDR/fetal liver kinase, Flk-1) first identified in 1991 [4], is produced within the cell and expressed on the cell surface as a matured 230 kD form (between 200–250 kD) of protein pending on levels of glycosylation [5]. In an intact cell, VEGFR2 binds certain members of the VEGF family [6] through dimerization and strong ligand-dependent tyrosine phosphorylation, which results in a mitogenic, chemotactic, and pro-survival signal [7]. VEGFR2 serves as the principal receptor for VEGF signaling [8] that leads to vasodilatation, endothelial cell migration, and proliferation [9]. VEGFR2-KO mice are embryonic lethal (at E8.5–9.5) with defective blood-island formation and vasculogenesis suggesting that VEGFR2 signaling is required for cardiovascular development [10]. Cell migration signals are recently shown to use, at least partly, a pathway dependent on an adaptor region of VEGFR2 [11]. Endothelial cells respond to VEGF to produce new blood vessels. This angiogenic process makes a critical contribution during embryogenesis and in the response to ischemia in adult tissues [12], [13], [14], [15]. VEGF resistance has been recently observed in diabetic angiogenesis which is attribute to monocytic VEGFR1 down-regulation [16]. The observation suggests that components or downstream targets of VEGF signaling, such as VEGFR2, could be missing or dysfunctional in diabetes. In fact, VEGFR2 protein reduction has been observed in patients with diabetes [17], [18] and in experimental diabetic animals [19]. The mechanism underlying VEGFR2 reduction and the contributions to angiogenesis impairment in diabetes are not known.

Methylglyoxal (MGO) is the major source of intracellular advanced glycation end-products (AGEs) [20]. It is a highly reactive α-oxoaldehyde being formed primarily from the intermediates of glycolysis in cells [21]. MGO has been implicated in the pathogenesis of diabetic complications [22]. Consistent with the finding that high glucose increases MGO production in cell culture *in vitro* [23], hyperglycemia enhances MGO production in patients with diabetes [24]. MGO can be detoxified efficiently by Glyoxalase (Glo) 1 [25]. While overexpression of Glo1 inhibits AGEs formation in cultured endothelial cells [26] and in diabetic animals [27], Glo1 deficiency is associated with increased intracellular AGEs [28]. Moreover, it has been reported that AGEs attenuate the angiogenic response *in vitro* [29]. In contrast, overexpression of Glo1 reverses high glucose-impaired angiogenesis in cultured endothelial cells [30]; blockade of AGEs formation by aminoguanidine restores ischemia-induced angiogenesis in peripheral limbs of diabetic mice *in vivo* [31]. Provided the crucial role of VEGFR2 in endothelial angiogenesis [32] and the implications of MGO in diabetic complications [22], this study investigated the impacts of MGO on VEGFR2 protein levels and endothelial angiogenesis in cell culture and mouse models to define a potentially new mechanism underlying angiogenesis impairment in diabetes.

RETRACTED

## Materials and Methods

### Materials

The antibodies used in the present study included: VEGFR2 (55B11), β-actin, Beclin-1, LC3B, SOD1, and peroxidase conjugated secondary antibodies (Cell Signaling, Danvers, MA); VEGFR2 (Flk-1:A-3), Bcl-2, Bax, Caspase 3, and Glo1 (Santa Cruz Biotechnology, Santa Cruz, CA); SOD2 (Fisher scientific, Pittsburgh, PA). The reagents included: MGO (Santa Cruz Biotechnology, Santa Cruz, CA); MG132 and mito-TEMPO-H (Enzo Life Sciences, Farmingdale, NY) (mTempol); protease inhibitor cocktail (EMD Chemicals, San Diego, CA); chloroquine, bafilomycin A1, pepstatin A, L-NAME, methotrexate (MTX), MTT, peroxynitrite, rapamycin, and uric acid (Fisher scientific, Pittsburgh, PA); ProLong® Gold and SlowFade® Gold Antifade Reagents and goat anti-rabbit IgG conjugates labeled with fluorescent dyes (Invitrogen, Carlsbad CA); epoxomicin, lactacystin, and z-VAD-fmk (Sigma, St. Louis, MO); SiRNA of human LC3B, Beclin-1,Receptor for AGE (RAGE), or control (Santa Cruz Biotechnology, Santa Cruz, CA); Adenoviral vectors expressing GFP, SOD1 or SOD2 (Vectors BioLabs, Philadelphia, PA); transfection-ready plasmids pCMV-Glo1 and pCMV-catalase, as well as their control DNA plasmids pCMV-GFP (OriGene, Rockville, MD).

### Endothelial Cells and Infection with Adenovirus, Plasmid, and siRNA

The endothelial cells: bovine aortic endothelial cells (BAEC) and human umbilicus vessel endothelial cells (HUVEC) cells and mediums were from ATCC (Manassas, VA). The cells were grown at 70–80% confluent and used between passages 3 and 8 as previously reported [33], [34], [35]. Adenoviral infection of GFP, SOD1, and SOD2 were performed as previously reported [35]. Confluent endothelial cells were infected with transfection-ready plasmid encoding Glo1 (pCMV-Glo1) or catalase (pCMV-catalase), as well as their control DNA plasmids (pCMV-GFP) according to instructions provided by OriGene (Rockville, MD). Transfection of pCDNA3 control or Beclin-1 was performed as previously described [36]. The plasmid vector pCDNA3-Beclin 1 was kindly provided by Dr. Junying Yuan through Addgene (Cambridge, MA: Addgene plasmid 21150). Transfection of control or target (LC3B, Beclin-1, and Glo1) siRNA was performed based on protocols provided by Santa Cruz Biotechnology (Santa Cruz, CA). All cells were incubated in a humidified atmosphere of 5% CO_2_+95% O_2_ at 37°C.

RETRACTED

### Western Blot Analysis

Cultured cells or aortas were homogenized on ice in cell-lysis buffer. Aortic VEGFR2 was detected through an immunoprecipitation-combined Western blot, where VEGFR2-co-immunoprecipitates were detected by Western blot with an antibody recognizing another VEGFR2 epitope. Western blotting and band densitometry were performed as previously reported [33], [34].

### Cell Viability Measurement

Endothelial cells were seeded at a density of 5×10^4^ cells/ml in 96-well plates. After being treated with MGO at studied concentrations, cell viability was measured using the MTT assay as previously reported [37]. Briefly, the cells after MGO or vehicle treatment were incubated with MTT (5 mg/ml, culture medium) and followed by absorption measurement at 490 nm. The cell viability was presented as a percentage of the DTT counts of the vehicle-treated cells.

### Cell Migration Assay

Cell migration was measured as previously reported [38]. Briefly, BAEC were plated at confluence and the monolayer artificially wounded by scraping with a pipette tip, followed by wash with medium and incubation with the studying reagents. Phase contrast cell images were taken after healing overnight. The wound healing was quantified by measuring the wounding area using the NIH ImageJ Program and expressed as percentage of the section area.

### Tube Formation Assay

The tube or vascular-like structure formation by endothelial cells was assessed on growth factor-reduced Matrigel (BD Biosciences), as described [39]. Briefly, endothelial cells were seeded on Matrigel-coated 24-well plates at 1×10^5^ cells per well in 1% FBS medium containing MGO or other reagents and incubated at 37°C for 18 hours. Tube formation images were observed using an inverted phase contrast microscope, and the degree of tube formation was quantified by measuring the number of tubes in 30 randomly selected fields quantified by the NIH ImageJ Program and expressed as a percentage of the total number of sprouts in control.

RETRACTED

### Quantification of MGO-modified Proteins (Adducts)

The quantification of MGO-modified proteins (MGO-protein adducts) was determined with an enzyme immunoassay kit (OxiSelect™ Methylglyoxal ELISA Kit) purchased from Cell BioLabs Inc. (San Diego, CA). This was accomplished by comparing the absorbance with that of a known MGO-bovine serum albumin standard curve according to the product manual provided by the manufacture.

### RNA Isolation, Reverse Transcription, and Real-time PCR

Total cellular RNA was isolated from endothelial cells, reverse transcribed into cDNA, and the resulting cDNA was subjected to quantitative polymerase chain reaction (PCR) as previously described [40]. Forward and reverse specific primer sequences were: VEGFR2 [40], forward: 5′-TGTGGGTTTGCCTAGTGTTTCT; reverse: 5′-CACTCAGTCACCTCCACCCTT. β-actin (75 bp, Human) primer: Forward: 5′-ACGGCATCGTCACCAACTG; reverse: 5′-GAGCCACACGCAGCTCATT. Total RNA Kit I (#R683401) was purchased from Omega Bio-Tek (Norcross, GA), iScript™ cDNA Synthesis Kit (170-8891), iQ™ SYBR Green Supermix (170-8880), and the Real Time Detection System were obtained from Bio-Rad (Hercules, CA). PCR specific primers were synthesized by Sigma (St. Louis, MO).

### Autophagy Assays (Confocal Microscopy of the Autophagosome)

Autophagy was visualized in endothelial cells by transfection of the plasmid pGFP-LC3 followed by analysis with confocal microscopy (Olympus FV500: Japan). The plasmid vector pGFP-LC3 was kindly provided by Dr. Toren Finkel through Addgene (Cambridge, MA: Addgene plasmid 24920). The autophagy assays were performed as previously described [41]. The number of GFP-LC3 punctae was assessed from >6 random high-power fields, and a minimum of 30 cells per sample were counted. An LC3 punctae was regarded as an isolated GFP-positive structure >1 µm diameter.

### Mouse Aortic Ring Assay

The assay was performed with aortic ring as previously described [42]. Briefly, thoracic aortas were excised from the mice, and peri-adventitial fibro-adipose tissues were removed. Aortas were then cut into 1-mm rings, washed in culture medium and transferred to 48-well tissue culture plates coated with Matrigel (100 µL per well), which was then overlaid with an additional 100 µL of Matrigel. The plates were incubated at 37°C, and media were changed every 2 days. MGO or other reagents were incubated with cell culture medium. Aortic rings were examined daily, and digital images were taken on day 6 for quantitative analysis of vascular endothelial outgrowth (sprouts) by the NIH ImageJ Program and expressed as a percentage of the total slide area per section.

RETRACTED

### Mice

Male C57BL/6J mice as well as genetic diabetic Akita and db/db (and control lean) mice, 8 weeks of age, 20–30 g, were obtained from the Jackson Laboratory (Bar Harbor, ME). Some groups of Akita mice were treated with mTempol (0.1 mM in the drinking water) or vehicle (normal drinking water) for 4 weeks. The animal protocols were reviewed and approved by the University of Oklahoma Institute Animal Care and Use Committee (IACUC). The approved IACUC protocol numbers are: 10-153-H, 11-072-H, and 11-045.

### Statistical Analysis

Values are expressed as mean ± SEM. All data were analyzed with 1-way ANOVA followed by multiple t-tests, except for those obtained by studies of time course and dose effects which were analyzed by repeated-measures ANOVA. Significance was accepted at *P*<0.05.

## Results

### MGO Reduces VEGFR2 Protein Levels and Impairs Endothelial Cell Migration and Tube Formation

We sought to investigate if MGO affected the protein levels of VEGFR2 in BAEC. First, we tested this in a range of MGO concentrations which have been widely reported. The results showed that incubation of MGO with endothelial cell reduced VEGFR2 protein levels in a time (Fig. 1A) and dose (Fig. 1B) dependent manner. The same dose and time effects of MGO were also observed in HUVEC (data not shown). Therefore, the lowest effective MGO concentration on VEGFR2 protein levels was defined as 25 µM overnight (16 h) under normal cell culture condition.

**Figure 1:** MGO reduces VEGFR2 protein levels and impairs endothelial cell angiogenesis. A and B: MGO reduced VEGFR2 protein levels in a time and dose dependent fashion. BAEC were incubated with MGO at indicated concentrations for up to 24 h. Then cells were subjected to Western blot respectively with a rabbit derived VEGFR2 antibody and a mouse derived β-actin antibody. All blots shown are representative of three independent experiments. *P<0.05 vs control (n = 3). C and D: MGO reduced endothelial cell angiogenesis in a dose dependent manner. Cells incubated with MGO (10–100 µM) were subjected to angiogenesis assessment by endothelial cell tube formation (upper panel in C) and migration (bottom panel in C). *P<0.05 vs control (n = 3).

To test the physiological outcome of the VEGFR2 reduction, we assessed angiogenesis, which was evaluated by assays of tube formation and cell migration in BAEC. In parallel with VEGFR2 protein reduction (Fig. 1A/B), the presence of MGO reduced tube formation (Fig. 1C, upper panel) and cell migration (Fig. 1C, bottom panel) in a dose-dependent fashion (Fig. 1D).

### MGO at the Studied Concentrations do not Affect Cell Viability and Markers of Apoptosis

MGO has been estimated to be produced to a level as high as 400 µM per cell per day [43], and similar concentrations have been applied in many physiological studies in literature. However, it is also well known that MGO at high concentrations induces cell death [44]. To decide whether MGO at the studied concentrations either altered the viability or induced cell apoptosis, we performed an MTT assay and examined apoptotic markers. As depicted in Fig. 2, there was no significant difference of viability between the control and MGO-treated cells at the studied concentrations of MGO (Fig. 2A). MGO at the indicated time course did not induce apoptosis of the treated cells, evidenced by no significant changes in Western blot staining for Bcl-2, Bax, and caspase 3, the classic markers of apoptosis (Fig. 2B).

RETRACTED

**Figure 2:** Knockdown of Glo1 enhances VEGFR2 reduction induced by MGO, whereas Glo1 overexpression prevents the reduction. A–B: MGO did not affect cell viability or apoptotic markers. BAEC were incubated with MGO at the indicated concentrations (for 24 h) or time course (up to 24 h) followed either by viability measurement (MTT assay) or Western blot staining for markers of apoptosis with respective antibodies against Bcl-2, Bax and Caspase 3. C: Knockdown of Glo1 by siRNA partly mimicked the MGO effect and enhanced MGO-induced VEGFR2 reduction. Transfection of control or Glo1 siRNA was performed based on protocols provided by Santa Cruz Biotechnology (Santa Cruz, CA). D: MGO increased levels of MGO-protein adduct which were further enhanced by siRNA knockdown of Glo1. E: Overexpression of Glo1 blocked MGO-induced VEGFR2 reduction. Infection of either control or Glo1 containing plasmid DNA was performed according to the protocol provided by OriGene (Rockville, MD). F: Overexpression of Glo1 blocked MGO-increased MGO-protein adducts. G: Knockdown of RAGE by siRNA prevented MGO-induced VEGFR2 reduction. Transfection of control or RAGE siRNA was performed based on protocols provided by Santa Cruz Biotechnology (Santa Cruz, CA). Western blot was performed with indicated antibodies. All blots shown are representative of three independent experiments. *P<0.05 vs control (n = 3). NS: not significant vs control (at 0 µM of MGO). Casp-3: Caspase-3; c-Casp-3: cleaved Caspase-3.

### Inhibition of Glo1 Enhances VEGFR2 Reduction Induced by MGO, whereas Overexpression of Glo1 Prevents the Reduction

To confirm that MGO generated its effect through a physiological pathway and that it was MGO specific, we monitored the effect of MGO in intact cells with either loss-of-function or gain-of-function approach that modulates Glo1, the MGO detoxifying enzyme [44]. In this regard, we first pre-incubated the cells with MTX, a Glo1 inhibitor [45] that increases MGO levels [46], before MGO-challenging. As shown in Fig. S1, the presence of MTX alone decreased VEGFR2 protein levels, mimicking the effect of MGO (Fig. S1); such an effect was enhanced in the presence of exogenous MGO where VEGFR2 protein levels were further decreased (Fig. S1). To exclude potential off-target effects of MTX, we employed a genetic approach with siRNA to knockdown Glo1 protein levels (Fig. 2C). Like MTX, Glo1 siRNA, but not the control, reduced VEGFR2 protein levels (Fig. 2C). The reduction was further enhanced when MGO was present (Fig. 2C). To further confirm that the effect was MGO-specific, we quantified the levels of MGO-protein adduct in the treated cells by ELISA. As depicted, MGO vs control increased intracellular MGO-protein adducts (Fig. 2D). Knockdown of Glo1 alone elevated MGO-protein adducts (Fig. 2D); such an effect was dramatically strengthened in MGO-treated cells (Fig. 2D). Next, we infected the cells with a Glo1-containing plasmid, using the cells infected with an empty plasmid as control. In line with the previous results (Fig. 1A/B, 2C and Fig. S1), MGO reduced VEGFR2 protein levels in the control cells (Fig. 2E); however, the reduction was absent in Glo1-overexpressing cells (Fig. 2E). Similarly, MGO augmented MGO-protein adduct levels in the control-plasmid but not the Glo1-overexpressing cells (Fig. 2F). Finally, we asked whether the effect of MGO required RAGE, the receptor for AGE. We choose to check VEGFR2 protein levels after the RAGE was knockdown. As expected, the RAGE protein staining was reduced in RAGE- but not control-siRNA treated cells (Fig. 2G). Importantly, the otherwise reduction of VEGFR2 was markedly prevented (around 80%) when RAGE was knockdown (Fig. 2G), suggesting a dominant role of RAGE in the studied effects of MGO. In sum, these data suggest that the MGO-generated effects were indeed physiologically relevant.

RETRACTED

### Inhibition of Autophagy, but not Proteasome or Caspase, Abolishes MGO-induced VEGFR2 Protein Reduction

To dissect the potential mechanism underlying VEGFR2 protein reduction, we measured VEGFR2 protein levels in the presence of proteolytic inhibitors. To this end, we pre-incubated BAEC with respective inhibitors of lysosome or autophagy, proteasome and caspase, prior to MGO challenge. As shown in Fig. 3A, pre-incubation with chloroquine (CQ), a widely recognized inhibitor for autophagy and lysosome, prevented VEGFR2 protein reduction. Other lysosome/autophagy inhibitors, such as pepstatin A (Pep A) (Fig. 3B) and bafilomycin A1 (Baf A1) (Fig. 3C) showed similar protective effects. To confirm the role of autophagy, we examined the effects of MGO in BAEC where important autophagy effectors, such as Beclin-1 and LC 3B [47], were knocked down. As presented in Fig. 3, MGO reduced VEGFR2 protein levels in the control-siRNA-infecting BAEC, as anticipated (Fig. 3D); however, Beclin-1 siRNA infection decreased Beclin-1 protein levels (Fig. 3D) and prevented VEGFR2 protein reduction by MGO (Fig. 3D). Similar VEGFR2-rescuring effects were observed when LC 3B was knocked down (Fig. S2). However, respective pre-incubation with MG132, epoxomicin, and lactacystin, the structurally unrelated inhibitors of proteasome, could not block the reduction (Fig. 3E), although VEGFR2 can be a proteasome target [48]; pre-incubation with z-VAD-fmk (z-VAD), a broad caspase inhibitor, also did not prevent the reduction (Fig. 3E). Next we wondered whether MGO affected VEGFR2 at the transcriptional level. To answer this question, we performed RT-PCR to quantify the mRNA levels of VEGFR2 in the presence of MGO. As shown in the Fig. S3, MGO at indicated time and dose did not change VEGFR2 mRNA levels; similar results were obtained in other settings where Glo1 was manipulated (Fig. S3). The data suggested that the effect of MGO mainly occurred at a protein level and that autophagy played a key role in MGO-mediated VEGFR2 reduction.

**Figure 3:** Inhibition of autophagy, but not proteasome or caspase, abolishes the reduction of VEGFR2 protein levels and angiogenesis by MGO. A–E: Suppression of autophagy, but not proteasome and caspase, prevented VEGFR2 reduction induced by MGO. (A–C and E) One hour prior to MGO challenge (25 µM for 16 h), BAEC were pre-incubated respectively with chloroquine (CQ: 100 µM), pepstatin A (Pep A: 10 µM), bafilomycin A1 (Baf A1: 5 nM), MG132 (0.5 µM), epoxomicin (Epo: 0.5 µM), lactacystin (Lact: 1 µM), and z-VAD-fmk (z-VAD: 20 µM); (D) Before MGO treatment (as above), BAEC were transfected either with control siRNA or siRNA targeting Beclin-1, based on instructions from Santa Cruz Biotechnology (Santa Cruz, CA); all cell lysates were subjected to Western blot with indicated antibodies. All blots shown are representative of three independent experiments. *P<0.05 vs control (n = 3). F: Administration of autophagy inhibitor rescued MGO-impaired tube formation. One hour before MGO stimulation (25 µM), endothelial cells were incubated respectively with CQ (100 µM), Pep A (10 µM), Baf A1 (5 nM) and subjected to tube formation assay. G: Knockdown of Beclin 1 by siRNA prevented MGO-reduced tube formation. All images presented are representative of three independent experiments. *P<0.05 vs control (n = 3). NS: not significant vs control.

### Autophagy Suppression Rescues MGO-impaired Endothelial Cell Tube Formation

To determine the physiological consequence of VEGFR2 protein restoration, we monitored endothelial cell tube formation with and without the presence of autophagy inhibitors. As demonstrated in Fig. 3, respective administration of CQ, Pep A and Baf A1 reversed the impaired tube formation (Fig. 3F), which was associated with restored VEGFR2 protein levels (Fig. 3A/B/C). However, application of the inhibitors alone did not affect endothelial tube formation (Fig. S4). Furthermore, the potential off-target effect of the inhibitors could be excluded, since the siRNA knockdown of Beclin 1 also rescued MGO-impaired endothelial tube formation (Fig. 3G), which was accompanied with restored VEGFR2 protein levels (Fig. 3D). All these data indicated the essential contribution of autophagy to the MGO-elicited effects.

RETRACTED

### MGO Increases Markers of Autophagy and Autophagic Flux, whereas Autophagy Induction Mimics the MGO-effects in Endothelial Cells

To further confirm the involvement of autophagy and exploit the underlying mechanism, we first measured protein levels of Beclin-1 and LC 3B, two common markers of autophagy [47], in MGO treated BAEC. As shown in Fig. 4, MGO increased both Beclin-1 and LC3B (mainly the LC 3B-II) protein levels (Fig. 4A). Of note, the increase in LC3B-II protein levels implicated an augmented conversion of LC3B-I to LC3B-II, a hallmark of autophagy in mammalian cells [49]. Next, we assayed the autophagic flux by counting the “LC3-dots or punctae” [50], a marker of autophagy initiation or autophagosome formation [49], [50]. As noted in the confocal imaging of the GFP-LC3 transfected cells (Fig. 4B), the MGO-treated cell presented a significant increase in number of LC3 punctae compared to untreated control (Fig. 4B), which was accompanied by an increase in autophagy markers (Fig. 2A). Furthermore, in VEGFR2-immuno-coprecipitates, the protein staining of LC3B-II was stronger in MGO challenged cells than the control (Fig. 4C), suggesting VEGFR2 as a potential target of autophagy. In agreement with this, genetic overexpression of Beclin 1 by plasmid infection reduced VEGFR2 protein levels without MGO (Fig. 4D), and the reduction was further enhanced with MGO (Fig. 4D). Finally, we explored whether pharmacological induction of autophagy exerted the same effect as MGO. We treated the cell with rapamycin, a well documented autophagy inducer [49]. As shown in Fig. 4E, this autophagy inducer decreased both VEGFR2 protein levels (Fig. 4E) and endothelial tube formation (Fig. 4F) in the absence of MGO. Taken together, these data indicated that autophagy was involved in VEGFR2 reduction induced by MGO.

RETRACTED

**Figure 4:** MGO induces autophagy markers and autophagic flux, whereas genetic or pharmacological induction of autophagy mimics MGO-elicited effects. A: MGO increased autophagy markers Beclin 1 and LC3B. B: MGO induced LC3 punctae formation (autophagic flux) (Confocal microscopy imaging). C: MGO increased immunoprecipitation of VEGFR2 with LC3B, an autophagy marker and a component of the autophagosome. D: overexpression of Beclin 1 decreased VEGFR2 protein levels, and the reduction was accelerated when MGO was present. E: Rapamycin (1 µM for 1 h) decreased VEGFR2 protein levels. F: Rapamycin (1 µM) reduced endothelial tube formation. BAEC were incubated with MGO (25 µM) for 1 h (A–C) and 16 h (D). Cells were collected for Western blotting with a rabbit derived Beclin-1 or LC 3B antibody and a mouse derived β-actin antibody. All blots shown are representative of three independent experiments. *P<0.05 vs control (n = 3).

### Suppression of Peroxynitrite Generation Prevents MGO-increased Markers of Autophagy in Endothelial Cells

Emerging data suggest that generation of reactive oxidative species (ROS), an important etiological factor for diabetic vascular complications [51],_ENREF_10 might trigger autophagy [52]. We wondered if the MGO-mediated effects involved peroxynitrite (ONOO^−^), one of the most important components of ROS [53]. ONOO^−^ is formed during simultaneous generation of superoxide (O_2_^–^.) and NO in a cell; inhibition of O_2_^–^ or NO abolishes ONOO^−^ formation [54]. As such, we incubated BAEC either with mito-TEMPO-H (mTempol) (a mitochondria-targeted antioxidant with O_2_^–^. scavenging properties [55]), L-NAME (a non-selective inhibitor of eNOS), or uric acid (UA) (a potent scavenger of ONOO^−^), before MGO stimulation. As shown in Fig. 5, mTempol treatment blocked the increase of Beclin-1 (Fig. 5A). Similarly, the increase was abolished either with L-NAME (Fig. 5B) or UA (Fig. 5C), an approach that suppresses ONOO^−^ formation. To further demonstrate the mediation by ONOO^−^, we monitored the expression of autophagy markers in ONOO^–^treated cells. As expected, ONOO^−^ incubation in the absence of MGO increased both Beclin 1 and LC3B protein levels peaking at 2 h (Fig. 5D). These data suggested that the MGO-induced autophagy was ONOO^−^ dependent and inhibition of ONOO^−^ generation inhibited autophagy induced by MGO.

**Figure 5:** MGO increases markers of autophagy through ONOO ^−^ **generation.** A–C: The MGO-increased autophagy marker (Beclin 1) could be prevented by blocking ONOO^−^ formation. BAEC were incubated respectively with mTempol (1 mM for 1 h), L-NAME (1 mM for 1 h), and UA (100 µM for 1 h) prior to MGO (25 µM, 1 h) incubation. D: ONOO^−^ per se induced both autophagy markers. BAEC were incubated with ONOO^−^ (100 µM) for up to 8 h. Cells were collected for Western blotting with a rabbit derived Beclin-1 (or LC3B) antibody and a mouse derived β-actin antibody. All blots shown are representative of three independent experiments. *P<0.05 vs control (n = 3). NS: not significant vs control.

RETRACTED

### Blocking ONOO^−^ Formation Abrogates MGO-mediated Reduction of VEGFR2 Protein Levels and Endothelial Cell Tube Formation

We wondered if inhibition of ONOO^−^ mimicked the effects of autophagy suppression which was shown to restore VEGFR2 protein levels (Fig. 3A/B/C) and endothelial angiogenesis (Fig. 3F/G). In this regard, we monitored VEGFR2 protein levels in the presence of ONOO^−^ suppression which was achieved with pharmacological or genetic means. We found that pre-incubation with mTempol restored VEGFR2 protein levels (Fig. 6A) in BAEC. Similarly, the reduction was abolished either by L-NAME (Fig. 6B) or UA (Fig. 6C). However, administration of mTempol, L-NAME, or UA alone did not affect endothelial tube formation (Fig. S4). Adenoviral overexpression of either SOD1 (Fig. 6D) or SOD2 (Fig. 6E), but not the control (GFP) (Fig. 6D/E), also blocked VEGFR2 reduction (Fig. 6D/E). Furthermore, the impaired endothelial angiogenesis appeared to be normalized, since a restored tube formation was evident when ONOO^−^ suppression through different mechanisms was present (Fig. 6F).

**Figure 6:** Suppression of ONOO ^−^ **generation prevents reduction of VEGFR2 protein and endothelial cell angiogenesis by MGO.** A–E: Suppression of ONOO^−^ generation prevented reduction of VEGFR2 protein. BAEC were incubated respectively with vehicle (controls), mTempol (1 mM for 1 h), L-NAME (1 mM for 1 h), and UA (100 µM for 1 h), adenoviral infection of GFP (control), or SOD1 and SOD2, prior to MGO incubation (25 µM, 16 h). The treated cells were subjected to Western blot for VEGFR2 protein. All blots shown are representative of three independent experiments. *P<0.05 vs control (n = 3). F: Inhibition of ONOO^−^ generation normalized the tube formation. Endothelial cells were incubated respectively with vehicle (controls), mTempol (1 mM for 1 h), L-NAME (1 mM for 1 h), and UA (100 µM for 1 h) prior to MGO challenge (25 µM). The treated cells were subjected to tube formation assay. The images shown are representative of three independent experiments. *P<0.05 vs control (n = 3). NS: not significant vs control.

Hydrogen peroxide is an important member of the reactive oxygen species and a regulator of endothelial function [56]. To decide whether hydrogen peroxide mediated the effects exerted by MGO, we compared these effects in cells overexpressing either a control (GFP) or an enzyme called catalase that catalyzes hydrogen peroxide degradation. As shown in Fig. S5, MGO reproducibly decreased both VEGFR2 (Fig. S5A) and endothelial tube formation (Fig. S5B). However, overexpression of catalase (Fig. S5A) could not prevent the reductions (Fig. S5A and S5B).

RETRACTED

### MGO Induces VEGFR2 Reduction in Endothelial Cell Cytosol which can be Blocked by Administration of Either O_2_^–^. Scavenger or Autophagy Inhibitor

VEGFR2 trafficking has recently been found to be associated with its function and stability [14], [57], [58]. We sought to detect VEGFR2 distributions in BAEC. As depicted in Fig. 7A/B (low/high power field), immune-fluorescent staining of VEGFR2 was found more in cytosol than in the cell membrane. MGO incubation reduced the staining in cytosol and membrane. However, pre-incubation of either mTempol or CQ restored the staining of VEGFR2 protein levels (Fig. 7B/C). In any cases, the nuclear VEGFR2 staining is not evident (Fig. 7A/B), although a functional nuclear localization of VEGR2 is recently characterized with reporter assays [59].

**Figure 7:** MGO induces endothelial VEGFR2 reduction predominantly in cytosol, which can be prevented by administration of O_2_^–^. scavenger or autophagy inhibitor. A–B (low and high-power fields of the same slides): MGO reduced VEGFR2 immune-staining in cytosol or cytoplasm membrane, without affecting staining in the nucleus. BAEC were incubated with MGO (25 µM, 16 h) and subjected to cell immunofluorescent staining with a commercial immune-staining kit including ProLong® Gold and SlowFade® Gold Antifade, by using a rabbit derived VEGFR2 antibody or stained with DAPI, and a goat anti-rabbit IgG conjugate labeled with fluorescent dyes. All images shown are representative of three independent experiments. C: The quantification results of B. *P<0.05 vs control (n = 3). NS: not significant vs control.

### Incubation of MGO with Mouse Aortas *ex vivo* Reduces Angiogenesis, which can be Abolished by Autophagy Suppression

To replicate the findings from cell culture study in a more physiologically relevant setting, we first performed *ex vivo* experiments in which the aortic rings from normglycemic mice (C57BL/6J) were challenged with MGO, with or without autophagy suppression and subjected to angiogenesis assessment by aortic ring assays. As presented in Fig. 8, MGO vs vehicle treated aortas manifested decreased capillary-like endothelial outgrowth (Fig. 8A); however, in the presence of either Pep A or Baf A1, the endothelial outgrowth was significantly restored (Fig. 8A), suggesting that autophagy mediated the MGO-reduced angiogenic response in aorta.

RETRACTED

**Figure 8:** VEGFR2 protein levels and the aortic endothelial angiogenesis are reduced in diabetic mice, which can be rescued either by autophagy suppression or O_2_^–^. scavenging. A: Aortic angiogenic response was reduced in MGO-challenged aortas of C57BL/6J mice, which could be restored by autophagy inhibitors. Aortic rings removed from normoglycemic C57BL/6J mice were incubated with MGO (25 µM) with or without the presence of autophagy inhibitors (Pep A: 10 µM, Baf A1: 5 µM) and subjected to aortic ring assay; *P<0.05 vs the vehicle treated (n = 5/group). B: Aortic endothelial outgrowth was impaired in db/db vs genetic control mice that could be rescued by autophagy inhibitors. Aortic rings prepared from the genetic control and db/db mice were treated with vehicle or autophagy inhibitors (Pep A: 10 µM, Baf A1: 5 µM) and followed by aortic ring assay. *P<0.05 vs the vehicle treated (n = 5/group). C–D: Aortic angiogenesis and VEGFR2 protein were reduced in diabetic Akita vs genetic control mice, which could be improved by mTempol administration *in vivo*. Aortas prepared from the genetic control and the treated Akita mice (mTempol: 0.1 mM in the drinking water, vehicle: normal drinking water, for 4 weeks) were subjected to aortic ring assay and aortic VEGFR2 protein detection by immune-precipitation (VEGFR2 enrichment)-combined Western blot. # indicates antibody recognizing different epitope of the VEGFR2 molecule. The Western blot of β-actin in aortic tissue homogenates with a mouse derived antibody is used as an Input for the loading control. *P<0.05 vs the vehicle treated (n = 5/group). E: the proposed mechanism of diabetic angiogenesis impairment: MGO, a glycolytic metabolite which is found to be increased in patients with diabetes, impairs endothelial angiogenesis through ONOO^–^dependent autophagy-mediated VEGFR2 degradation. NS: not significant vs control.

### Aortas of Genetic Diabetic Mice Present Autophagy-mediated Lower Angiogenic Response Compared to the Genetic Controls

We next examined whether aortas from the genetic diabetic db/db and Akita mice had lower angiogenic capacity and whether that could be reversed through autophagy inhibition. To this end, we assessed angiogenesis of the aortas from db/db and the genetic control mice with or without autophagy suppression. As depicted in Fig. 8, aortas from db/db vs the control mice presented reduced aortic endothelial outgrowth (Fig. 8B); similar blunted angiogenic responses were also observed in another type of genetic diabetic Akita mice (Fig. 8C). However, pre-treatment either with Pep A or Baf A1 normalized the endothelial outgrowth (Fig. 8B), indicating the involvement of autophagy in angiogenesis impairment in diabetes.

RETRACTED

### Administration of mTempol *in vivo* Prevents the Reduction of VEGFR2 Protein Levels and Restores Aortic Angiogenic Response in Akita Mice

We took one step further to determine if administration of mTempol *in vivo* rescued aortic angiogenic capacity through VEGFR2. To achieve this, we treated the Akita mice either with mTempol (0.1 mM, in drinking water) or vehicle (normal drinking water) for 4 weeks and assessed the angiogenic response and VEGFR2 protein levels of the aortas. As shown in Fig. 8C, mTempol treatment *in vivo* improved aortic endothelial outgrowth (Fig. 8C). With a VEGFR2 enrichment approach, we were able to detect aortic VEGFR2 proteins of non-diabetic genetic control mice (Fig. 8D), which were reduced in Akita mice (Fig. 8D). However, administration of mTempol, but not of the vehicle, restored the aortic VEGFR2 protein levels (Fig. 8D). In summary, diabetes impaired endothelial angiogenic capacity appeared to be associated with VEGFR2 protein levels, both of which could be normalized by administration of mTempol, a scavenger of O_2_^–^.

## Discussion

The present study provided evidence to demonstrate that MGO, a glycolysis metabolite found increased in patients with diabetes, impairs endothelial angiogenesis both in cell culture and aortic tissues. This is operative through ONOO^–^dependent and autophagy-mediated VEGFR2 degradation, because pharmaceutical and genetic approaches that inhibit either autophagy or ONOO^−^ formation reverse the MGO-mediated impacts. Importantly, the same approaches both *ex vivo* and *in vivo* restored the angiogenic response or VEGFR2 protein levels in diabetic aortas, suggesting a previously unidentified mechanism for angiogenesis impairment in diabetes (Fig. 8E).

Angiogenesis impairment in diabetic peripheral vasculature contributes to delayed wound healing, increased risk of rejection of transplanted organs, exacerbated peripheral limb ischemia, and even cardiac mortality [2], [60]. However, the mechanisms underlying diabetes-impaired angiogenesis are not completely understood. A growing body of evidence support that AGEs, as well as MGO, the major precursor of AGEs, and the receptor of AGEs (RAGE) are implicated in the pathogenesis of diabetic vascular complication [61]. MGO is believed to contribute to diabetic complications either as a direct toxin or as a precursor for advanced glycation end products. Consistent with this notion, the present study has implicated an important role of RAGE (Fig. 2G) and the MGO-detoxifying system (Fig. 2E) for MGO-generated effects. Indeed, it has been demonstrated that AGE restriction may improve angiogenesis and wound healing in diabetic animal model [62]. The relevance of AGEs-altered angiogenesis can also be seen in MGO-impaired gastric ulcer healing [63]. Recently, it has been found that O-GlcNAc modification mediated-Akt inhibition reduces angiogenesis [64] and that the Akt-pathway also mediates the AGEs-effects on angiogenesis [65]. However, the dependency of Akt-pathway is lost pending serum presence, and it is yet to establish what serum factor contributes to the observations [65]. Nevertheless, these data imply that other factors essential in the angiogenic pathway are involved. For instance, the alterations of VEGFR1 have been shown to contribute to the impaired angiogenesis after hindlimb ischemia in a type 2 diabetic mouse model [66]. In current study, we have not been able to detect as significant changes of the VEGFR1 as those of the VEGFR2 (data not shown).

RETRACTED

Given the crucial role of VEGFR2 in endothelial angiogenesis [67], [68], [69], [70], downregulation of endothelial VEGFR2 protein demonstrated in the present study could be a new mechanism. Surprisingly, quantitative data of VEGFR2 protein in aortic tissues are few in literature, in contrast to those reported either in cultural endothelial cells or in the circulation. One plausible reason could be that endothelial VEGFR2 expression in normal vascular tissue is low [71]. Indeed, only by immunoprecipitation enrichment could we detect VEGFR2 protein in control aortic tissues and its reduction in diabetes (Fig. 8D). In endothelia cells, VEGFR2 is found localized in endothelial caveolae, associated with caveolin-1, and this complex is rapidly dissociated upon stimulation with VEGF [72]. A recent study showed that a significant amount of VEGFR2 exists in endosome [15] and undergoes constitutive endosome-to-plasma membrane recycling [73]. The MGO-induced VEGFR2 reduction identified in the present study occurred predominantly in cytosol (and may be in plasma membrane as well). The observation implicates that MGO-mediated VEGFR2 degradation could be a detour from its normal trafficking. Such a deviation might represent an unidentified cellular mechanism by which diabetes reduces VEGR2 protein levels. Although the role of trafficking in MGO-mediated VEGFR2 reduction remains to be established, the alteration of VEGFR2 protein immune-fluorescent-staining in the presence of MGO and the involvement of both ONOO^−^ and autophagy (Fig. 7A/B/C) were confirmed with other approaches (Fig. 1–6 and Fig. 8A/B/C). Furthermore, aortic rings from diabetic (Akita and db/db) vs genetic control mice demonstrated lower angiogenic capacities (Fig. 8C/D), which were associated with VEGFR2 protein reductions (Fig. 8D). More importantly, the clinical relevance of VEGFR2 reduction in diabetes is apparent in that diabetes-associated VEGFR2 reductions have been observed both in humans [17], [18] and experimental animals [19]. It is believed that such reductions impair collateral formation in the myocardium of patients with diabetes [17], [18] or causes erectile dysfunction in the penile of diabetic rats [19].

RETRACTED

To the best of our knowledge, this is the first report that links autophagy-mediated VEGFR2 degradation to angiogenesis impairment in diabetes. The supporting evidence not only includes the induction of autophagy markers (Fig. 4A and 5A/B/C: LC3B and/or Beclin-1) but also the pharmacological (Fig. 3A/B/C and Fig. 4E/F: experiments with autophagy/lysosome inhibitors or inducer) and genetic (Fig. 3 D/G and Fig. S2/Fig. 4D: experiments with siRNA or overexpression) connections of autophagy to the reductions of VEGFR2 (Fig. 3A/B/C/D, Fig. 4D, and Fig. S2) and angiogenesis (Fig. 3F/G and Fig. 4F). The key evidence included the demonstration of MGO-enhanced autophagy initiation (increase in the number of LC3 punctae) (Fig. 4B) and immune-coprecipitation of LC3B with VEGFR2 (Fig. 4C). Importantly, induction of autophagy either mimicked (Fig. 4D) or enhanced the MGO-generated effects (Fig. 4D/E/F). These data suggest that VEGFR2 is a potential target of autophagy. Autophagy is a lysosomal degradation pathway and essential for survival, differentiation, development, and homeostasis [47]. The pathway refers to a regulated catabolic cellular process for the lysosomal-dependent turnover of organelles and proteins [74]. Autophagy principally plays an adaptive role to protect organisms against diverse pathologies, including infections, cancer, aging, heart disease, and neurodegeneration. However, in certain disease settings, self-eating or even the pro-survival functions of autophagy could be deleterious [47]. Although emerging evidence supports the role of autophagy in the pathophysiology of diabetes, especially in the maintenance of pancreatic function, it remains largely undecided whether autophagy plays a protective or harmful role in other organ-tissue systems [75], [76]. Interestingly, several angiogenesis inhibitors employed in anti-angiogenesis therapy induce autophagy activation [77], [78], linking autophagy initiation to angiogenesis suppression [79]._ENREF_41 Consistently, suppression of autophagy apparently promotes angiogenesis [79]. Indeed, mice deficient in the autophagic protein Beclin-1 display a pro-angiogenic phenotype associated with hypoxia [80]. Therefore, an autophagy-mediated reduction of VEGFR2 may contribute to diabetic angiogenesis impairment. Evidence in this paper also supports an ONOO^−^ dependent mechanism regulating autophagy and its effects, consistent with the recognized role of oxidative stress in diabetic complications [24]. However, it merits further investigations on how autophagy is triggered to reduce VEGFR2. Due to the heterogeneity of angiogenic dysregulation in diabetes [3] and the fact that angiogenesis is determined by a range of factors beyond vascular cell [81], it remains to be elucidated if VEGFR2-associated proteins or other angiogenic-related factors in vascular cell and beyond [82] would be affected by similar mechanism under diabetic conditions.

RETRACTED

Provided the important role of VEGFR2 in angiogenesis [67], [68], [69], [70] and the association of AGEs/precursors (including MGO) with the pathogenesis of diabetic complications [22], [83], [84], [85], we propose that impaired physiological angiogenesis in diabetes results, at least in part, from downregulation of VEGFR2. Mechanistically, MGO reduces endothelial cell angiogenesis through ONOO^−^ dependent and autophagy-mediated VEGFR2 protein degradation, which may represent a potentially new mechanism for angiogenesis impairment in diabetes.

## Supporting Information

Figure S1 **Administration of Glo1 inhibitor mimics the effect of MGO and accelerates MGO-induced VEGFR2 reduction.** BAEC were pre-incubated with Glo1 inhibitor MTX (100 µM for 1 h) followed by MGO administration at 25 µM for 16 h. Cell homogenates were subjected to Western blot with a rabbit derived VEGFR2 antibody and a mouse derived β-actin antibody. All blots shown are representative of three independent experiments. *P<0.05 vs control (n = 3).
(JPG)

Figure S2 **LC3B knockdown prevents VEGFR2 reduction in MGO-treated endothelial cells.** BAEC were transfected either with control siRNA or siRNA targeting LC3B, according to instructions from Santa Cruz Biotechnology (Santa Cruz, CA). Then the cells were challenged by MGO (25 µM for 16 h) and the cell lysates were subjected to Western blot with indicated antibodies. All blots shown are representative of three independent experiments. *P<0.05 vs control (n = 3). NS: not significant vs control.
(JPG)

Figure S3 **MGO does not change mRNA levels of VEGFR2.** A: MGO did not alter mRNA levels of VEGFR2. BAEC were incubated with MGO at indicated representative (1X and 2X) concentrations (1×25 µM, which was used through the present study; 2×25 µM) for up to 8 h. B: Manipulation of Glo1 by administration of Glo1 inhibitor did not change VEGFR2 mRNA levels. BAEC were pre-incubated with of Glo1 inhibitor MTX (100 µM for 1 h) followed by MGO administration at 25 µM for 16 h. All cells from A and B were subjected to total cellular RNA isolation (Total RNA Kit I: #R683401, Omega Bio-Tek), reverse transcription into cDNA (iScript™ cDNA Synthesis Kit, #170-8891, Bio-Rad), and quantitative polymerase chain reaction (PCR) (iQ™ SYBR Green Supermix, 170-8880 and Real Time Detection System, Bio-Rad). The mRNA levels of VEGFR2 were normalized with those of the actin mRNA. NS: not significant vs control (n = 3).
(JPG)

Figure S4 **The studded reagents do not alter endothelial tube formation.** BAEC were pre-incubated respectively with chloroquine (CQ: 100 µM), pepstatin A (Pep A: 10 µM), bafilomycin A1 (Baf A1: 5 nM), mTempol (1 mM), L-NAME (1 mM), and UA (100 µM) for 1 h, and then all were subjected to assay of endothelial tube formation. All images presented are representative of three independent experiments. NS: not significant vs control (n = 3).
(JPG)

Figure S5 **Overexpression of catalase does not prevent MGO-induced reduction of VEGFR2 protein levels and endothelial cell tube formation.** HUVEC were transfected with pCMV control (GFP) or catalase (CAT)-expressing plasmid, according to instructions from OriGene (Rockville, MD). The transfected BAEC were incubated with MGO (25 µM for 16 h) and then subjected to A: Western blot. B: tube formation assay. All images or blots shown are representative of three independent experiments. *P<0.05 vs control (n = 3). CAT: catalase. NS: not significant vs control (n = 3).
(JPG)
